# Early Detection of Medical Image Analysis by Using Machine Learning Method

**DOI:** 10.1155/2022/3041811

**Published:** 2022-02-23

**Authors:** Ahmad M. Khasawneh, Amal Bukhari, Mahmoud Ahmad Al-Khasawneh

**Affiliations:** ^1^Department of Cybersecurity, Amman Arab University, Amman 11953, Jordan; ^2^College of Computer Science and Engineering, University of Jeddah, Saudi Arabia; ^3^School of Information Technology, Skyline University College, University City Sharjah, 1797 Sharjah, UAE

## Abstract

We develop effective medical image classification techniques, with an emphasis on histopathology and magnetic resonance imaging (MRI). The trainer utilized the curriculum as a starting point for a set of data and a restricted number of samples, and we used it as a starting point for a set of data. As calibrating a machine learning model is difficult, we used alternative methods as unsupervised feature extracts or weight-conditioning factors for identifying pathological histology pictures. As a result, the pretrained models will be trained on 3-channel RGB pictures, while the MRI sample has more slices. To alter the working model using the MRI data, the convolutional neural network (CNN) must be fine-tuned. Pretrained models are placed and then used as feature snippets. However, there is a scarcity of well-done medical photos, making training machine learning models a difficult endeavor to begin with. In any case, data augmentation aids in the generation of sufficient training samples; however, it is unclear if data augmentation aids in the prediction of unknown data samples. As a result, we fine-tuned machine learning models without using any additional data. Furthermore, rather than utilizing a standard machine learning classifier for the MRI data, we created a unique CNN that uses both 3D shear descriptors and deep features as input. This custom network identifies the MRI sample after processing our representation of the characteristics from beginning to end. On the hidden MRI dataset, our bespoke CNN outperforms traditional machine learning. Our CNN model is less prone to overfitting as a result of this. Furthermore, we have given cutting-edge outcomes employing machine learning.

## 1. Introduction

In the era of medical healthy recognition of histopathology for cells and tissues under the microscope used in this study, these complement each other in the performance of life functions. Recently, medical image analysis takes a long time to analyze. Therefore, the interpretation of hidden medical experts about the interpretation of images or samples is not rare. In addition, samples can be diagnosed with the help of the computer (CAD), which is considered by medical experts as a high balance that helps in conducting local diagnoses. Therefore, the medical pathologist begins by taking a biopsy of the living tissue [1]. As the biopsy that was examined and then through which the tissue is removed. The tissue removed from the organ is placed in a fixative before being examined under a microscope. To be able to differentiate between the different cellular levels under the microscope, tissues are usually stained for ease of work and precision and tissues are stained with hematoxylin and eosin (H&E). Then, the pathologist examines the tissue slide to learn their findings according to their experience. To be able to apply computational techniques, tissue slides must first be digitized [2]. Therefore, digitizing histological slides should be either as micrographs (i.e., containing a single disease condition) or as a whole slide image (WSI) (i.e., usually containing multiple disease areas).

X-rays are used by specialized devices that help diagnose the disease and in several ways, including magnetic resonance (MRI) [3] to create an image of the particular organ with the technique of generating a magnetic field and thus drawing the outputs of those rays [4]. Here comes the role of the computer to draw an illustration in black and white with multiple levels for each specific time, and as a group of images, they are treated in a complex manner Figure 1.

Medical images are considered one of the most popular practices recently, as their presence in digital form for building CAD applications for image processing/analysis techniques [5]. Linking different medical images using machine learning (ML), which can be categorized as moderated or unsupervised ML, is one of the most prominent topics currently. In the case of supervised learning, we train a model on a set of images where the base truth label is known. Several supervised learning algorithms that are widely known in the literature on medical image classification are to be used: as in Multilayer Perception (MLP) [6], Support Vector Machine (SVM) [7], and others. On the other hand, in the absence of base truth labels, unsupervised learning which is designed to find out hidden patterns can be adopted through a mapping function, for example, means aggregation or Principal Component Analysis (PCA) [8].

Our goal is to develop, apply, and comparatively evaluate techniques that are capable of actively and evidently classifying medical images.

This model was created by developing a multitrainable machine learning technique capable of performing classification tasks using traditional texture-based features [9].

Therefore, in this paper, we use the basis of shearlet positive classification techniques for Alzheimer's patients. The Alzheimer's Disease Neuroimaging Initiative (ADNI) database and the Open Access Imaging Studies Series (OASIS) are used to attain this purpose [10].

As mentioned previously, machine learning suffers from computer costs and a lack of laboratory equipment, through the lack of tests on which machine learning depends to obtain a feature vector for each chip that will represent the magnetic resonance imaging sample. To solve these problems in Alzheimer's disease, we adjust machine learning with a model that has the ability to create cognitively relevant recipes to encode characteristics of Alzheimer's disease and differentiate it from other cognitive diseases, in order to take advantage of feature space generation through the capabilities of the CNN model to learn feature maps from the slices for a more efficient stack of the MRI sample [11].

We suggest investigating the integration of both 3D and shearlet descriptor features. After the feature vector sequences are computed from the shearlet, the domain CNN model, we propose to train a classification model in the following: (1) classic classifier training (SVM and DTB) and (2) building a custom CNN model for vector end-to-end postprocessing features [12].

## 2. Related Work

Alzheimer's disease (AD) is critical for a pathologist to suggest appropriate treatment for patients. Different methods are used with the pathological tissue classification process. Therefore, we use techniques for visual, gray-level texture-based repetition matrix, variable-scale feature transformation, local binary pattern, and gradient histogram [13]. Besides that, features that depend on texture are extracted from a whole image or at least the specific section in the image like gray matter, brain spinal, or white matter. Since GLCM comes, four descriptors can be obtained: variance, correlation, homogeneity, and energy. As a result, just a portion of some slides is run in the training, while the vector of features will not be averaged if all segments are used [14].

The author suggested many steps for a new diagnosis of the acute lymphoblastic leukemia approach. This method entails acquiring blood images using the public dataset (ALL-IDB1), segmenting blast cells using marker-based segmentation (MBS), and then extracting features from segmented blast cells using the gray level cooccurrence matrix (GLCM) with reduced and selected specific features using probabilistic main component analysis. Furthermore, Random Forest (RF) was introduced to categorize the segmented cell into the normal or abnormal group at the classification level [15].

Additionally [16], there are three important classes of classification with the following: AD vs. CN, pMCI vs. CN, and pMCI vs. sMCI. Next, descriptors from PCA used in the training mode in the SVM classifier depend on extracted features with reducing samples of MRI. The Fisher Discrimination Ratio (FDR) scores were used to arrange the PCA descriptors in descending order. Also, in terms of extracting information from the return on investment, there are several studies that have been worked on by some researchers. For instance, the authors computed cooccurrence matrices from voxel coupling [17].

These characteristics were derived from various MRI scan locations, including the hippocampus, precuneus, and posterior cingulate cortex. GLCM was employed instead of tissue-based spatial domain slices to implement this method.

However, there are several methods that have been used in the field of magnetic resonance imaging data in terms of several different measurements, analyses, and guidelines [18]. Each MRI slice was transformed using a double complex wavelet transform tree (DTCWT). The PCA was used to reduce the wavelet coinage clients. To distinguish CN samples from AD samples, forwarding neural networks were used. Likewise [19], the Daubechies wavelet (DW) was utilized to convert each MRI image into directions and power subbands; after that, a construct of descriptors is used, and for nearest neighbors, AD classification is suggested.

The shearlet transform was used which has really anisotropic waveforms, which in previous studies were based on size only [20], where coins are used to classify decorative images, for example [21]. Shearlet-based descriptors were used by fairing to judge images. While building local power features of shearlet coins, quantifying and encoding these local power features make it represent it as a fixed rotation. And in all energy graphs for all levels of decomposition, the backlog represents the properties of the image [22]. It has been suggested that there are specific levels of bronchial field decomposition of breast tumor ultrasound in classifying the images.

An approach was proposed for textured image classification and retrieval, using linear regression where the dependencies of adjacent shearlet subdomains are modeled to represent classification subshearlet domains, to compute the power descriptors. However, the image retrieval is hermetic by both the stats in the contour and the shearlet domains [23], as shown in Figure 2.

## 3. Shearlet-Based Training in Machine Learning

In order to implement the histopathological image as used in AD, we apply training classifiers to the complex shearlet transform and with the complex coefficients compute the magnitude and relative phase (RP), as shown in Figure 3.

The shearlet transform, used for image classification as the authors explain, is an effective tool for capturing two-dimensional orientation features from an image. However, the shearlet coefficients for the spatially distributed discontinuities must be specified and are in contrast to the constants [24], although curves and contours have similar characteristics to cuts within certain constraints [25]. A curvelet was created based on the rotation operator. Do not maintain the digital network, as subsistence lacks solid theory [26]. On the other hand, the property of the shearlet transform is its use of shear to control directional selectivity. This process does not destroy the digital network, that is, unlike curvelet transformation which happens in most cases. Therefore, shearing is allowed digital implementation of the shearlet transform. The shearlet transform depends on the affine system theory. There are three operators in this affine system as follows:

1. First, the dilation operator that is based on the parabolic scaling *A*_*a*_ matrix, where *a* > 0:

(1) $$\begin{array}{c} A_{a=}\left(\begin{array}{cc} a & 0\\ 0 & a^{1/2} \end{array}\right) \end{array}$$

(2) Second, to capture the orientations of waveforms, the shearing matrix *B*_*s*_ is utilized, where *s* € *R*:

(2) $$\begin{array}{c} B_{s=}\left(\begin{array}{cc} 1 & s\\ 0 & 1 \end{array}\right) \end{array}$$

(3) Finally, a translation operator (*t* € *R*2) is used to change the position

To obtain the shearlets in the discrete domain [27], the continuous shearlets are sampled on a discrete set of parameters. As such, one can choose *a* = 2^−*j*^ and *s* = −1, where *j*; *l* € *Z*, to compute *M*_2−*j*,−1_. Then, *M*2_*M*_2−*j*,−1__^ −1^*M*_2*j*,1_= *B*^*l*^*A*^*j*^, where *B* and *A* can be known as

(3) $$\begin{array}{c} A_{=}\left(\begin{array}{cc} 4 & 0\\ 0 & 2 \end{array}\right),\\ B_{=}\left(\begin{array}{cc} 1 & 1\\ 0 & 1 \end{array}\right). \end{array}$$

Given that *j*; *l* € *Z* and this translation parameter *t* is replaced with *k* € *Z*2, the discrete shearlet transform then can be obtained as

(4) $$\begin{array}{c} \Psi_{j,l,k}\left(x\right)=\left|detA\right|\frac{i}{2}\;\Psi \left(B^{i}A^{j}x-k\right). \end{array}$$

There are a set of new samples that capture the statistical distribution/information of the shearlet size/stage components for each scale and trend after this complex shearlet transformation computation [28]. The magnitude and phase coefficients of a complex number *C* = *a* + *ib*, where *a* is the real component and *b* is the imaginary part, are defined as $P=\sqrt{a^{2}+b^{2}}$ and *θ* = tan^−1^(*b*/*a*), straight. However, a comparison with others who use or take into account only the magnitudes since the efficacy of these treatments for their stage and their ability to classify biomedical images is important with its ability to classify biomedical images.

However, to categorize tight pictures, [29] relied on extracting descriptors from the relative phase (RP) of a sophisticated vectorial filter bank. Therefore, the relative stalk phase coefficients are extracted. The complex shearlet transform with *S* scales and *K* orientations for each scale decomposes a given image of size *N* *N*. The subband phase angle coefficient at position *I* *j*) at scale *s* and orientation *k* is denoted as _(*sk*) (*i*, *j*), where *s* = 1, 2, ⋯, *S* and *k* = 1, 2, ⋯, *K*. *S* = 4 and *K* = 8 per scale in our study.

The RP of a directional subband is calculated as follows for a given phase coefficient at position *I* *j*):

(5) $$\begin{array}{c} {\text{RP}}_{ak}\left(i,j\right)=\left\{\begin{array}{cc} \theta_{ak}\left(i,j\right)-\theta_{ak}\left(i,j+1\right), & \text{if }1\leq k\leq \frac{k}{2},\\ \theta_{ak}\left(i,j\right)-\theta_{ak}\left(i+1,j\right), & \text{if }\frac{k}{2}\leq k\leq K. \end{array}\begin{array}{c} \;\\ \; \end{array}\right. \end{array}$$

The complex shearlet transformation was implemented in ShearLab. Therefore, the vertical and horizontal differences were selected due to the shear direction of the shear transformation. However, the multiscale, omnidirectional shearlet transform provides multiresolution analysis of textured images. Moreover, achieving the computation of statistical descriptors for each directional subdomain (size and RP) is important in the implementation phase [30].

## 4. Method and Discussion

Methodology mainly consists of four stages starting with the preprocessing stage that is responsible for image preparation like noise reduction then extracting new useful features from an image to provide for the next stage of classification by certain classifiers, and the last stage has to evaluate the proposed result to benchmark with existing results.

### 4.1. Proposed Model and Components

Figure 4 depicts the model for our proposed project. The fusion of both deep features and shearlet descriptors is worthy here in the proposed study. The proposed system comprising two MRI samples and pipelines is preprocessed in the first step of our study, as indicated in the picture. The shearlet transform coins are then summed up using some important procedures, as each summarization differs from one way to another in supporting a useful set in descriptors of MRI samples so that the gain of high-end performance is achieved. When using the ADNI dataset, descriptors of SFTA will classify correctly. As a result, for the OASIS dataset, the cooccurrence matrix synthetic features produced the best classifier.

The use of CNN variables is extracted from MRI utilization samples, and the use of updating models is in terms of features [31]. Simulated results show that SVM classification is achieved compared with other techniques such as the SoftMax layer. As a result, SoftMax was used to try in the proposed research. By training the traditional ML class, the features were utilized separately. However, we found that the deep MobileNet features extracted by OASIS in addition to ASNI datasets achieved worthy results during classification. Finally, the suggested descriptors might be bound by these methods:

1. For the classic class, both shearlet-based feature and ML are fed in the system
2. The proposed CNN model was also fed by combining both deep features and descriptor of shearlet. Then, system components were outlined in detail

The neural network is the main component of machine learning designed to adapt with progress needed; it consists of three parts including the input layer (which are features extracted from images), output layers (which are predicted evaluated results), and hidden layer considered the intermediate layer that is adaptive with the process in terms of the number of layers and node numbers in such layer as shown in Figure 5.

#### 4.1.1. The 3D Shearlet Transform

Samples of MRI have different sizes such as *a*, *b*, and *c* attached with *S* scales of directions *K* in each 3D scale for shearlet transform in data of MRI. For convolution with the MRI specimen, the holographic dimension of liters, *a* *b* *z*, is employed. A structure of dimension *a* *b* *c* *z* serves as the foundation for this arrangement, with *a*, *b*, *c*, and *z* denoting height, breadth, number of slats, and meters, respectively. We get the average presence of all shearlets after collecting the volume of coins for each segment with varied orientations; thus, the *I* segment is defined by only one mean shearlet subdomain (for example, *a* × *b* × *i* × 1). The severe devaluation of the shearlet coins is important. Otherwise, it will end up with too many descriptors per slice while computing the features derived from the direction of each subband. In addition, manipulating whole descriptors of segmented MRI samples through a trait vector results in a high number of features within less training [32].

The rating results are low for news samples due to the overfitting of the rating tool. Therefore, an attribute representation can be obtained for the average stories of the segment *I* slice in one vector *d*_*i*_ = (*d*^1^, *d*^2^, ⋯, *d*^3^), where *j* represents the length of the vector. However, the MRI sample of the latter feature vector may be referred to as *F* = (*d*_1_, *d*_2_, ⋯, *d*_*n*_), such that *n* is considered the MRI samples.

#### 4.1.2. Shearlet-Based Descriptors

The different descriptors are inconsistent with each other through the extended feature, which combines the different shearlet descriptors to help it improve its performance. Thus, there is a set of features that take certain specific aspects of the descriptors that were used jointly to the advantage of the individual descriptors and the ability to achieve reasonable accuracy. So, we do the following fusion test:

Fusion 1: descriptors of shearlet magnitude or RP (CM+LBP+LOSIB+SFTA)

Fusion 2: shearlet magnitude or RP descriptors (CM+LOSIB)

Fusion 3: shearlet magnitude coefficients (CM+LBP+SFTA+CM Dot) and shearlet RP coefficients (CM+LBP+LOSIB) [33]

### 4.2. CNN as Feature Extractor

In the task of classifying breast cancer tissue images, the use of a pretrained model combined with logistic regression as a classifier resulted in good classification results. Four pretrained CNN models capable of handling the complexity of MRI datasets were employed in this study: SqueezeNet-v1.1 [34], MobileNetv2 [35], Inception-v3 [36], and Xception [37].

For the proposed study, we aim to use samples of MRI in different channels which we stack the slides deeply. Thus, each CNN-certified model must be modified in such way.

Modify the input layer, *h* *w* *c*, by modifying the dimensions of the magnetic resonance imaging sample, by making the channel number (*c*) of MRI greater than three. This includes a pretrained input layer similar to RGB images, as well as a convolution layer adjacent to the input layer on a pretrained array of weights with channel size = 3. As a result, it should replace this convolution layer with the new input layer's channel size and train them from the beginning.

Furthermore, certain layers such as the pool and convolution layer in addition to the dense layer run in the training mode with a certain dataset before proceeding with the testing mode and increase the features by filtering the image sample; then, because the dataset we are working with is binary, we need two dimensions for the classification layer.

We have mentioned in prior studies magnetic resonance imaging samples. As a result, modifications to machine learning, pretrained by the latest technologies in knowledge networks and features of the stacked MRI sample, are being implemented at the same time. As a result, each model employed in this study has a description and features, such as the following:

- SqueezeNet-v1.1 contains 8 modules, which are Fire2-Fire9. Each unit has 2 expansion layers, one with a size of 1 × 1 core and one with a size of 3 × 3. However, feeding both expansions into the depth chain layer leads to a definition of the size *a* × *b* × *c* per unit by creating feature maps. In this form, we select the “Fire9” module. We are working on an average of each feature map that generates a feature vector with a size of 1 × 1 × *c*, so the mapping vector of features in MRI is considered
- Also, the MobileNet.2 is made up of 16 blocks and is divided into two types: a linear bottleneck process and a skip connection. The following procedures are found in both blocks: convolution, batch normalization, and the modified linear unit (ReLU). As a result, min(max(*x*, 0), 6) is added to ReLU to limit the minimal output. The pooling layer (avg.) is output as the last layer in deep used in the proposed but first to the initialization layer
- Inception-v3 is a model that uses a unit that draws input data to several different branches where each branch links through channels with a set of convolutions of size 1 1. So, the treatment for this feature maps across another set of convolutions with ranks 3 3 or 5 5. As all of these feature maps are sequential, the output of Avg Pool is utilized as the deepest layer shortly before the classification layer in this model
- Xception is a model with 36 convolutional layers that are formulated in 14 pcs. So, it is based on a deep detachable wrap of the layers where only the first and last blocks have no residual connections around them, but the rest have a residual linear connection around them. It is similar to Inception-v3, which has an Avg Pool layer in this model

In this study, we look at the performance of two classifiers in particular. First, SVM is used for binary classification (one-to-one class judgments) [38]. We balance all feature vectors before training to ensure that they have the same mean and variance. The kernel function transforms the input data into a higher-dimensional feature extraction, which is then used to simulate the input tissue dataset's hyperlevel classification.

Second, each classifier in the set is a classification and regression tree, according to DTB (CART). The dataset is broken down using the decision tree. As a result, the dataset's inclusions are reduced with each partition when compared to the original dataset [39].

Therefore, we explore the following fusion of various deep features obtained under the supervision of the various ML models:

Fusion 1: (SqueezeNet (Fire9)+MobileNet (Avg Pool)+Xception (Avg Pool)+Incorporation descriptors (Avg Pool))

Fusion 2: MobileNet (Avg Pool)+Xception (Avg Pool)+Incorporation (Avg Pool) descriptors

Our use of our custom CNN model is to integrate manual descriptors and deep features. We examined the feature set exclusively within the same domain, thus either handcrafted descriptors together or deep features together. In this field, combining both handcrafted and fully deep features is our proposal in this work. Below is a comparison between the mergers as follows:

- All our extracted manual descriptors are in the form of a single data array that is aggregated (e.g., *A*) then spread with all features in deep (*B*); this is done for all MRI brain scans
- It is made up of a single collection of handcrafted descriptors and a single set of deep features (i.e., so each set is determined based on its performance as it is used individually). This fusion is only applicable to brain MRI data

Averaging of classified performance illustrate in

(6) $$\begin{array}{c} \text{ACC}=\left(\text{TP}+\text{TN}\right)=\left(\text{TP}+\text{TN}+\text{FP}+\text{FN}\right)=\left(\text{TP}+\text{TN}+\text{FP}+\text{FN}\right)=\left(\text{TP}+\text{TN}+\text{FP}+\text{FN}\right)=\left(\text{TP}+\text{TN}+\text{FP}+\text{FN}\right)=\left(\text{TP}+\text{TN}+\text{FP}+\text{FN}\right)=\left(\text{TP}+\text{TN}+\text{FP}+\text{FN}\right). \end{array}$$

- Positive represents the true positive ratio or can say *S* = TP + FN and also considered sensitivity (*S*)
- Negative represents the ratio of true negative then TN+FP refer to defining specificity (SP)
- $\text{GM }\left(\text{geometric mean}\right)=\sqrt{\text{Sen}\times \text{SP}}$

Our unique CNN models are constructed from the ground up, with 70% used for training and 40% used for validation, due to the time commitment of training machine learning models. The best-performing model is based on the availability of separate hidden data tested from start to finish using shearlet-based descriptors and classifiers.  Table 1 illustrates an example.

## 5. Results and Discussion

### 5.1. Results of Classification Utilizing Shearlet-Based Descriptors

The results of feature extraction using a shearlet-based model are presented in this paper. Nonetheless, Table 2 and Figure 5 illustrate DTB and SVM performance, on the ADNI and OASIS datasets used in this study. As a result, the classification results of the classifiers shown below are obtained using 5-fold nested cross-validation.

The OASIS dataset is used to test our 3D shearlet technology. As a result, when fed into a classification model utilizing the OASIS dataset, our approach obtains accuracy ranging from 76 to 81%, as shown in Figure 6. While classifying the dataset using the synthetic features of the cooccurrence matrix associated with a class SVM with a corresponding sensitivity of 0.6117, specificity of 0.7330, and geometric mean of 0.6614 yielding the highest accuracy of 0.8122, the merge boosts accuracy to 0.7002 when using the DTB model as shown in Table 2.

### 5.2. Achievement Results in Training Mode

CNN results are illustrated in Tables 3 and 4 by using extracted features on OASIS and ADNI datasets. For the ideal universe when utilizing the DTB model, the pretrained MobileNet leads to strong classification results when trained in a fivefold overlapping CV pattern for both datasets used in our investigation.

We also found that by using two distinct types of deep feature merging to classify both datasets (ADNI and OASIS), the classification results did not improve. The statistical significance of the *t*-test for MobileNet results against deep fusion of feature 2 to classify the ADNI dataset is not significant at *p* 0.05, where the *t* value and *p* value are 0.6631 and 0.2629 as illustrated in Figure 7. Similarly, by classifying the dataset of OASIS using a *t*-test of MobileNet performance against deep feature fusion 2, the result is not significant at *p* 0.05 with a *t* value of 0.8885 and a *p* value of 0.2001.

Descriptors and features illustrated in Tables 5 and 6 expose the shearlet-based feature set normal extracted features by DTB and SVM classifiers first shown in Fusion 1 with the ADNI dataset to achieve high accuracy. As a consequence, by picking only the best performance, the SVM model was employed to get the highest accuracy achieved by proposing two classifiers when trained in 5-fold CV using 80% to 40% for training and validation.

Therefore, the combination is used to train the OASIS. While using a DTB, we attain the highest classification accuracy of 80% by merging all features extracted with descriptors; the acquired classification accuracy is 82.88 percent (i.e., the ones that got the best accuracy on their own). As a result, this model was chosen to be tested using never-before-seen data (i.e., data that had been hidden from the start to the end). The proposed two classifiers in terms of 5-fold CV and CNN classifiers are trained with a training and validation ratio of 40% to 80%.

Classified images will be trained on the patient attributes or hidden data, as described earlier. As a result, the proposed approach can be used to detect AD brain scans in patients who are not all at the same stage of the disease.

## 6. Conclusion

The major purpose of this study is to develop a model for medical image classification that is both efficient and accurate. To that end, we have presented two pipelines, one that uses manual procedures based on clipping descriptors and the other that uses machine training methods. MRI scans, on the other hand, can be used to carefully design prescriptions and extract relevant information and features from the content of medical images. In addition to the difficulties in histopathology pictures, which employ magnetic resonance imaging, there are other issues to consider. Each sample contains a large number of 2D image slices. As a result, we will have to adapt our methods to deal with class cation MRI samples. As a result, using a three-dimensional shearlet transform, calculate a shearlet-based feature representation. We do not employ pretrained machine learning (CNN) models as unsupervised feature extractors, on the other hand, because we would have to feed each slice separately to generate a trait vector for each slice. As a result, we use the MRI samples to tweak a pretrained model, which we then employ as a feature extractor for the entire MRI sample.

Our shearlet-based descriptors are also linked to important Alzheimer's disease classification criteria. In addition, future work while reviewing our strategies may extend the descriptors suggesting new features by MI segmentation. It is important to look for a multimodal brain tumor image segmentation standard (BRATS), for example. Furthermore, some research has suggested that categorization models be built based on specific segments.

## Figures and Tables

**Figure 1:** Image analysis of MRI related to Alzheimer's disease by using ML [4].

**Figure 2:** Medical image fusion.

**Figure 3:** Shearlet transform domain.

**Figure 4:** Proposed model for 3D shearlet-based textural descriptors with ADNI and OASIS MRI classification features.

**Figure 5:** Construction of neural network.

**Figure 6:** Performance of OASIS descriptor performance.

**Figure 7:** Deep features improve ADNI classification efficiency.

**Table 1:** ADNI descriptor performance.

Technique		ACC	Sen	SP	GM
Fusion 1	SVM	0.8101	0.8740	0.6534	0.6801
	DTB	0.7052	0.7229	0.6771	0.7066
Fusion 2	SVM	0.6756	0.6448	0.6663	0.6792
	DTM	0.7052	0.7115	0.7000	0.7088

**Table 2:** OASIS descriptor performance.

Technique		ACC	Sen	SP	GM
Fusion 1	SVM	0.8652	0.7012	0.7620	0.6599
	DTB	0.7002	0.6229	0.7771	0.6966
Fusion 2	SVM	0.6556	0.5448	0.7663	0.6392
	DTM	0.7002	0.6115	0.7885	0.6888

**Table 3:** ADNI classification performance using deep features.

Technique		ACC	Sen	SP	GM
SqueezeNet	SVM	0.8602	0.9001	0.8218	0.8378
	DTB	0.8950	0.8774	0.9132	0.8939
MobileNet	SVM	0.9050	0.8948	0.9063	0.8987
	DTB	0.9100	0.9161	0.8964	0.9052
Xception	SVM	0.9000	0.8744	0.9217	0.8963
	DTB	0.9050	0.8839	0.9241	0.9021
Inception	SVM	0.8650	0.8861	0.8410	0.8631
	DTB	0.8800	0.8839	0.8727	0.8776
Fusion 1	SVM	0.8700	0.8756	0.8608	0.8665
	DTB	0.8800	0.8839	0.8727	0.8776
Fusion 2	SVM	0.8650	0.8661	0.8608	0.8622
	DTB	0.8800	0.8839	0.8727	0.8776

**Table 4:** Performance of OASIS of deep features.

Technique		ACC	Sen	SP	GM
(1) SqueezeNet	SVM	0.9123	0.8732	0.9214	0.8832
	DTB	0.8823	0.8677	0.9126	0.8861
(2) MobileNet	SVM	0.9157	0.9024	0.9387	0.9184
	DTB	0.9288	0.9156	0.9477	0.9291
(3) Xception	SVM	0.9010	0.9014	0.9085	0.9010
	DTB	0.8869	0.8919	0.8969	0.8894
(4) Inception	SVM	0.8859	0.9081	0.8773	0.8889
	DTB	0.9016	0.8966	0.9139	0.9023
Fusion 1	SVM	0.8829	0.9064	0.8843	0.8906
	DTB	0.9030	0.8976	0.9059	0.8975
Fusion 2	SVM	0.9020	0.9266	0.8823	0.9001
	DTB	0.9011	0.8956	0.9039	0.8975

**Table 5:** Performance of ADNI with proposed features.

Technique		ACC	Sen	SP	GM
(a) Descriptors without CNN					
Fusion 1	SVM	0.9120	0.9210	0.9210	0.8992
	DTB	0.8750	0.8900	0.8600	0.8742
Fusion 2	SVM	0.8750	0.9400	0.9300	0.9345
	DTB	0.8950	0.9100	0.8800	0.8933
(b) Descriptors with CNN					
Fusion 1	CNN	0.9002	0.8901	0.9050	0.9101
Fusion 2	CNN	0.9003	0.9003	0.9020	0.8992

**Table 6:** Combined performance of OASIS.

Technique		ACC	Sen	SP	GM
(a) Descriptors without CNN					
Fusion 1	SVM	0.8944	0.9000	0.8889	0.8922
	DTB	0.9000	0.9000	0.9000	0.8981
Fusion 2	SVM	0.9278	0.9111	0.9444	0.9274
	DTB	0.8944	0.8889	0.9000	0.8944
(b) Descriptor with CNN					
Fusion 1	CNN	0.8671	0.9021	0.8001	0.7983
Fusion 2	CNN	0.9500	0.9603	0.9302	0.9291

## Data Availability

Data are available upon request.
